# Predicting the impact of environmental factors on citrus canker through multiple regression

This article has been retracted.

**DOI:** 10.1371/journal.pone.0260746

**Published:** 2022-04-05

**Authors:** Akhtar Hameed, Muhammad Atiq, Zaheer Ahmed, Nasir Ahmed Rajput, Muhammad Younas, Abdul Rehman, Muhammad Waqar Alam, Sohaib Sarfaraz, Nadia Liaqat, Kaneez Fatima, Komal Tariq, Sahar Jameel, Hafiz Muhammad Zia Ullah Ghazali, Pavla Vachova, Saleh H. Salmen, Mohammad Javed Ansari

**Affiliations:** 1 Institute of Plant Protection, MNS-University of Agriculture, Multan, Pakistan; 2 Department of Plant Pathology, University of Agriculture, Faisalabad, Pakistan; 3 Department of Plant Breeding and Genetics, University of Agriculture, Faisalabad, Pakistan; 4 Institute of Molecular Biology and Biotechnology, The University of Lahore, Lahore, Pakistan; 5 Department of Biochemistry and Molecular biology, University of Gujrat, Gujrat, Pakistan; 6 Plant Pathology Section, Oilseeds Research Station, Khanpur, Pakistan; 7 Department of Botany and Plant Physiology, Faculty of Agrobiology, Food and Natural Resources, Czech University of Life Sciences Prague, Kamycka, Prague, Czech Republic; 8 Department of Botany and Microbiology, College of Science, King Saud University, Riyadh, Saudi Arabia; 9 Department of Botany, Hindu College Moradabad (Mahatma Jyotiba Phule Rohilkhand University Bareilly), Moradabad, India; Ghazi University Dera Ghazi Khan, PAKISTAN

## Abstract

Climatic conditions play a significant role in the development of citrus canker caused by *Xanthomonas citri pv*. *citri* (*Xcc*). Citrus canker is regarded as one of the major threats being faced by citrus industry in citrus growing countries of the world. Climatic factors exert significant impacts on growth stage, host susceptibility, succulence, vigor, survival, multiplication rate, pathogen dispersion, spore penetration rate, and spore germination. Predicting the impacts of climatic factors on these traits could aid in the development of effective management strategies against the disease. This study predicted the impacts of environmental variables, i.e., temperature, relative humidity, rainfall, and wind speed the development of citrus canker through multiple regression. These environmental variables were correlated with the development of canker on thirty (30) citrus varieties during 2017 to 2020. Significant positive correlations were noted among environment variables and disease development modeled through multiple regression model (Y = +24.02 + 0.5585 X1 + 0.2997 X2 + 0.3534 X3 + 3.590 X4 + 1.639 X5). Goodness of fit of the model was signified by coefficient determination value (97.5%). Results revealed the optimum values of environmental variables, i.e., maximum temperature (37°C), minimum temperature (27°C), relative humidity (55%), rainfall (4.7–7.1 mm) and wind speed (8 Km/h), which were conducive for the development of citrus canker. Current study would help researchers in designing better management strategies against citrus canker disease under changing climatic conditions in the future.

## Introduction

Citrus is one of the major fruit crops grown in >140 countries situated in tropical and subtropical regions of the world [1–7]. It is a popular fruit cultivated globally due to its easier availability, popularity, commercial importance, and a major source of vitamin C. It has a significant contribution towards human nutrition. The Citrus orchards are attacked by *Xanthomonas citri* pv. *citri* (*Xcc*), which is a noxious pathogen causing citrus canker disease [8–10]. *Xanthomonas citri* is a straight, rod shaped, mono-flagellum, gram-negative bacterium with a wide host range [11]. Citrus canker is one of the most notorious citrus diseases in Florida, USA, leading towards mass eradication of plants in the entire state [12]. The disease is still spreading even after spending an estimated 12 million US$ annually on its management [13–15]. The *Xcc* infestation initially seen as a small lesion on the leaves, which is expanded in later stages and ultimately become necrotic surrounded by water-soaked, oily margins. Chlorotic rings of yellow color appear on the surfaces of fruits, leaves and stems as disease progresses and these rings eventually develop into a crater-like appearance [6, 16]. The Asiatic citrus leaf-miner (*Phyllocnists citrella*) significantly accelerates the severity of citrus canker through feeding and transferring bacterium to new leaf growth [17].

The Environmental factors play a crucial role in the dispersion and multiplication of *Xcc*. The bacterium multiplies rapidly in the lesions and transfer to other plants under ample moisture availability [18]. Furthermore high rainfall and wind speed accelerate the dispersion rate of the disease [19]. Extreme weather conditions such as tropical storms and hurricanes result in long-distance dissemination of the pathogen and increase disease infestation [20–23]. Environmental factors significantly affect host susceptibility, succulence, vigor, survival, and multiplication rate of the pathogen, pathogen dispersion, and spore penetration and germination rates. Earlier studies indicated that temperature between 30–38°C with high relative humidity play a crucial role in the disease development [24, 25].

A couple of similar studies [26, 27] reported that temperature, wind velocity, relative humidity and rainfall are the main factors responsible for the spread and development of citrus canker disease. Strong wind driven rain splashes provided conducive environment for the dispersal of citrus canker [28–30]. Similarly, hot summer and mild winter with some alternations of low and high temperature make the pathogen more aggressive [31]. The *Xcc* multiplies in the lesions of leaves, stems, and fruits, and disperse to new healthier host plants by rain splashes. During the presence of ample moisture on lesions, the bacteria ooze out and disperse to infect new plant growth. Rainstorms during monsoon increase the epidemics of citrus canker in the presence of active source of inoculum [32, 33].

Climate anomalies are resulting in unstable conditions for plants’ growth since past years, which ultimately exert immense pressure on food production. The studies relating to epidemiological factors helps in management decisions by determining the conducive environmental conditions for the development of diseases such as citrus canker [34, 35]. Hence, development and utilization of disease predictive model with relation to environmental factors is probably the most effective way to manage the prevalence of citrus canker disease. However, unfortunately no such work has been previously done under the climatic conditions of Pakistan. Correlation of environmental variables in the prevalence and perpetuation of *Xcc* under native climatic conditions of the country has been computed and interpreted in this study. The results would provide novel perceptive to manage citrus canker disease under changing environmental conditions.

## Materials and methods

### Data collection

This three-year study collected citrus canker disease incidence data from the experimental area of Department of Plant Pathology, University of Agriculture Faisalabad, Pakistan. Data relating to environmental variables including maximum and minimum temperatures (°C), wind speed (Km/h), rainfall (mm) and relative humidity (%) were obtained from meteorological station located at Agronomy research area, University of Agriculture Faisalabad, Pakistan. The relationship of these environmental variables with the disease development was predicted by regression and correlation analysis and a predictive model was developed based on the obtained results.

### Regression analysis

Regression analysis was used to determine the relationship between environmental variables and disease development/incidence [36, 37]. Two different regression models, i.e., simple, and multiple regression models were used in the study. The mathematical equations for these models are presented as Eq 1 and Eq 2.


Y=β0+β1x (Eq 1)

Here, Y acts as response variable in case of disease, while X works as explanatory variable. The β0 denotes as intercept and β1 is the slope.

For multiple linear regression models, more than one explanatory or predictor variables (X) are included as compared to the simple linear regression analysis.


Y=β0+β1x1+β2x2+⋯+βixi+∈ (Eq 2)

Here, x characterizes the compilation of predictors x1, x2,… xi in the model, and β1, β2,…βi act for the corresponding regression coefficients and ∈ is the random error or interruption in the experiment [38, 39].

### Characterization of environmental factors conducive for citrus canker

All environmental data as well as disease incidence (%), and alterations in the environmental factors and disease incidence were analyzed by least significant difference test (LSD at P<0.05) [40]. The effect of environmental factors on citrus canker disease was modeled by correlation. Mean square error (MSE) Mallows Cp and R^2^ were used a criteria for selecting the best models [41, 42].

### Goodness of fit of the model

The correlation was used for determining the goodness of fit of the model [43–45]. The varieties/cultivars in which >50% of the environmental variables exerted significant effect were plotted and most conducive environmental factors for disease development were determined. The manipulation of these factors on disease infestation was tested by drawing a comparison between observed and predicted disease incidence values by multiple regression models [45, 46]. Furthermore, disease predictive model depending on environmental conditions was developed which has significant influence on citrus canker disease development.

### Statistical analysis

The data consisted of an average of three replicates and differences among treatments were estimated by one-way analysis of variance (ANOVA). The means were compared using least significant difference post-hoc test (P < 0.05) where ANOVA indicated significant differences. All statistical computations were made on SPSS 20.0 [47]. Microsoft excel 2016 was used to calculate the standard errors of the meas. Graphical presentation was completed on Origin Pro 9.0 (OriginPro, Northampton, USA). The minimal dataset of the study has been uploaded as S1 Dataset.

## Results

### Development and evaluation of citrus canker predictive model

Multiple regression equation of citrus canker predictive model for two years was Y = +24.02 + 0.5585 X_1_ + 0.2997 X_2_ + 0.3534 X_3_ + 3.590 X_4_ + 1.639 X_5_. Here (Y = disease incidence X_1_ = maximum temperature, X_2_ = minimum temperature, X_3_ = relative humidity, X_4_ = rainfall and X_5_ = wind speed). The R^2^ value expressed that model was statistically fitted well for environmental variables. Some data points deviated from the reference line according to the normal probability (Fig 1), while most values were scattered equally around the residual line in case of residual vs. fit model which showed better fit (Fig 2). Few data points were little far from the line of reference i.e., near to zero; -3.5 to + 4 primarily exhibited as an error in the regression model. Model was designed according to [36].

**Fig 1:** Plot of normal probability for the citrus canker disease predictive model based on two years data.

**Fig 2:** Residual versus fit plot for the regression model of citrus canker disease.

### Assessment of disease predictive model by comparing dependent variables with regression coefficient through physical theory

Analysis of variance of regression articulated that maximum and minimum temperature, relative humidity, rainfall, and wind speed significantly contributed towards disease development. The R^2^ value of 97.5% expressed that model was statistically suitable under given environmental conditions. Variable’s coefficients of regression model for citrus canker are given in Table 1.

**Table 1:** Regression model’s coefficients of variables for citrus canker disease.

Parameter	Coefficient	Stander Error	t-Stat	*P*-value
Intercept	-24.02	2.56	-9.40	0.000*
Maximum temperature (°C)	0.5585	0.0570	9.80	0.000*
Minimum temperature (°C)	0.2997	0.0302	9.92	0.000*
Relative humidity (%)	0.3534	0.0495	7.14	0.000*
Rainfall (mm)	3.590	0.319	11.26	0.000*
Wind speed (Km/h)	1.639	0.147	11.14	0.000*

* = Significant at *P*< 0.05.

### Estimation of model for predicted and observed values

For assessing the reliability of model, value differences of observed and predicted data points were estimated. Among observed values, fourteen data points were beyond reference line (standard error = 1.81517) and created an error in experiment. According to graphs, maximum prediction (464 out of 480 values) values have differences (less than 5) were consolidated between 95% confidence interval (C.I) and 95% predictive interval (P.I) which showed that there was a good fit between predictive and observed values (Fig 3).

**Fig 3:** A fitted line plot for citrus canker disease with observed and predicted data points at 95% confidence and predictive intervals.

### Correlation of environmental variables with the development of citrus canker disease on various citrus varieties during 2017–18 and 2018–19

Maximum and minimum temperature, relative humidity, rainfall and wind speed had significant positive correlation (P≤ 0.05) with citrus canker incidence during both years on thirty varieties (Blood red (*Citrus sinensis cv*. *blood red*), Malta (*Citrus reticulata cv*. *malta*), Mayer lemon (*Citrus limonia cv*. *mayer lemon*), China lemon (*Citrus limonia cv*. *china lemon*), Feutral’s early (*Citrus reticulate cv*. *feutral’s early*), Sweet lemon (*Citrus limettioides*), Jaffa (*Citrus sinensis cv*. *jaffa*), Succari (*Citrus sinensis cv*. *succari*), Mungal singh (*Citrus reticulata cv*. *mungal singh*), Grapefruit (*Citrus paradise*), Tangerine (*Citrus reticulata cv*. *tangerine*), Musambi (*Citrus sinensis*), Pine apple (*Citrus sinensis cv*. *pine apple*), Valentia late (*Citrus sinensis cv*. *valentia* late), Kinnow (*Citrus reticulata cv*. *kinnow*), Key lime (*Citrus aurantifolia*), Trifoliate orange (*Citrus poncirus*), Pomelo (*Citrus grandis*), Orange (*Citrus sinensis*), Bitter orange (*Citrus aurantium*), Rough lemon (*Citrus jambhiri*), Lemon (*Citrus limon*), Citron (*Citrus medica*), *Citrus paradise cv*. *foste*r, *Citrus paradise cv*. *duncan*, *Citrus paradise cv*. *shamber*, *Citrus sinensis cv*. *washington navel*, *Citrus sinensis cv*. *rubby red*, GAL GAL *(Citrus pseudolimon*), Persian lime (*Citrus latifolia*) (Tables 2 and 3).

**Table 2:** Pearson correlation matrix of various environmental factors with citrus canker disease on different citrus varieties during 2017–18.

Sr #	Variety Name	Max. T (°C)	Min. T (°C)	RH (%)	RF (mm)	WS (Km/h)
1	*Citrus sinensis* cv. *blood red*	0.768**	0.906**	0.945**	0.453**	0.812**
2	*Citrus reticulata* cv. *Malta*	0.758**	0.899**	0.949**	0.457**	0.821**
3	*Citrus limonia* cv. *mayer lemon*	0.713**	0.853**	0.971**	0.577**	0.781**
4	*Citrus limonia* cv. *china lemon*	0.765**	0.906**	0.945**	0.466**	0.813**
5	*Citrus reticulata* cv. *feutral’s early*	0.824**	0.942**	0.921**	0.477**	0.756**
6	*Citrus limettioides (Sweet lime)*	0.806**	0.920**	0.938**	0.468**	0.790**
7	*Citrus sinensis* cv. *Jaffa*	0.639**	0.774**	0.889**	_0.484_ _**_	0.706**
8	*Citrus aurantifolia swingle (Kagzi lime)*	0.559**	0.700**	0.930**	_0.494_ **	0.855**
*9*	*Citrus reticulata* cv. *mungal singh*	0.730**	0.818**	0.860**	0.451**	0.667**
*10*	*Citrus reticulata* cv. *Kinnow*	0.784**	0.928**	0.892**	0.493**	0.756**
11	*Citrus reticulata* cv. *Tangerine*	0.696**	0.790**	0.810**	0.297^Ns^	0.535**
12	*Citrus sinensis* cv. *Succari*	0.710**	0.865**	0.977**	0.515**	0.819**
13	*Citrus sinensis* cv. *pine apple*	0.687**	0.785**	0.807**	0.484**	0.621**
14	*Citrus sinensis* cv. *valentia late*	0.705**	0.858**	0.978**	0.546**	0.827**
15	*Citrus paradise*	0.781**	0.915**	0.934**	0.456**	0.809**
16	*Citrus aurantifolia (Key lime)*	0.446**	0.597**	0.865**	0.529**	0.833**
17	*Citrus poncirus (Trifoliate orange)*	0.661**	0.772**	0.896**	0.567**	0.823**
18	*Citrus grandis (Pomelo)*	0.558**	0.679**	0.895**	0.390^Ns^	0.740**
19	*Citrus sinensis*	0.761**	0.899**	0.952**	0.461**	0.817**
20	*Citrus aurantium (Bitter Orange)*	0.594*	0.662**	0.693*	0.301^Ns^	0.605**
21	*Citrus jambhiri (Rough lemon)*	0.757**	0.899**	0.952**	0.468**	0.814**
22	*Citrus medica (Citron)*	0.502**	0.584**	0.717**	0.352^Ns^	0.434**
23	*Citrus japonica (Kumquat)*	0.585**	0.682**	0.710**	0.565**	0.678**
24	*Citrus latifolia (Persian lime)*	0.430*	0.562**	0.817**	0.457**	0.730**
25	*Citrus pseudolimon (GAL GAL)*	0.661**	0.672**	0.619**	0.250^Ns^	0.518**
26	*Citrus sinensis* cv. *ruby red*	0.584**	0.735**	0.971**	0.510**	0.818**
27	*Citrus sinensis* cv. *washington navel*	0.435**	0.509**	0.620**	0.256^Ns^	0.514**
28	*Citrus paradise* cv. *Shamber*	0.792**	0.920**	0.941**	0.448**	0.786**
29	*Citrus paradise* cv. *Duncan*	0.761**	0.899**	0.952**	0.461**	0.817**
30	*Citrus paradise* cv. *Foster*	0.763**	0.902**	0.949**	0.448**	0.813**

The values are Pearson’s correlation coefficient

Ns = non-significant

* = significant (P <0.05)

** = Highly significant.

**Table 3:** Correlation of environmental factors with canker disease on different varieties of citrus for 2018–19.

Sr#	Variety Name	Max. T (°C)	Min. T (°C)	RH (%)	RF (mm)	WS (Km/h)
1	*Citrus sinensis* cv. *blood red*	0.619**	0.760**	0.945**	0.922**	0.796**
2	*Citrus reticulata* cv. *Malta*	0.608**	0.75**	0.949**	0.922**	0.799**
3	*Citrus limonia* cv. *mayer lemon*	0.509**	0.664**	0.949**	0.851**	0.805**
4	*Citrus limonia* cv. *china lemon*	0.561**	0.709**	0.964**	0.894**	0.821**
5	*Citrus reticulata* cv. *feutral’s early*	0.692**	0.814**	0.915**	0.921**	0.800**
6	*Citrus limettioides (Sweet lime)*	0.699**	0.802**	0.909**	0.886**	0.769**
7	*Citrus sinensis* cv. *Jaffa*	0.544**	0.658**	0.900**	0.832**	0.757**
8	*Citrus aurantifolia swingle (Kagzi lime)*	0.228**	0.421**	0.842**	0.804**	0.830**
9	*Citrus reticulata* cv. *mungal singh*	0.555**	0.653**	0.787**	0.786**	0.724**
10	*Citrus reticulata* cv. *Kinnow*	0.623**	0.772**	0.943**	0.937**	0.813**
11	*Citrus reticulata* cv. *Tangerine*	0.551**	0.676**	0.858**	0.880**	0.807**
12	*Citrus sinensis* cv. *Succari*	0.564**	0.654**	0.610**	0.572**	0.410**
13	*Citrus sinensis* cv. *pine apple*	0.684**	0.795**	0.922**	0.923**	0.783**
14	*Citrus sinensis* cv. *valentia late*	0.578**	0.734**	0.957**	0.935**	0.877**
15	*Citrus paradise*	0.655**	0.793**	0.930**	0.924**	0.791**
16	*Citrus aurantifolia (Key lime)*	0.378^Ns^	0.516**	0.839**	0.859**	0.831**
17	*Citrus poncirus (Trifoliate orange)*	0.747**	0.867**	0.827**	0.924**	0.728**
18	*Citrus grandis (Pomelo)*	0.649**	0.775**	0.935**	0.941**	0.844**
19	*Citrus sinensis*	0.687**	0.827**	0.898**	0.859**	0.789**
20	*Citrus aurantium (Bitter Orange)*	0.633**	0.747**	0.924**	0.880**	0.828**
21	*Citrus jambhiri (Rough lemon)*	0.613**	0.761**	0.945**	0.942**	0.808**
22	*Citrus medica (Citron)*	0.701**	0.788**	0.891**	0.835**	0.732**
23	*Citrus japonica (Kumquat)*	0.383^Ns^	0.531**	0.868**	0.863**	0.683**
24	*Citrus latifolia (Persian lime)*	0.703**	0.816**	0.899**	0.921**	0.827**
25	*Citrus pseudolimon (GAL GAL)*	0.369^Ns^	0.491**	0.741**	0.678**	0.666**
26	*Citrus sinensis* cv. *ruby red*	0.451**	0.613**	0.808**	0.835**	0.822**
27	*Citrus sinensis* cv. *washington navel*	0.553**	0.586**	0.649**	0.699**	0.635**
28	*Citrus paradise* cv. *Shamber*	0.678**	0.798**	0.910**	0.876**	0.771**
29	*Citrus paradise* cv. *Duncan*	0.631**	0.771**	0.943**	0.929**	0.815**
30	*Citrus paradise* cv. *Foster*	0.628**	0.765**	0.945**	0.924**	0.808**

The values are Pearson’s correlation coefficient

Ns = non-significant

* = significant (P <0.05)

** = Highly significant.

### Characterization of environmental factors conducive for the development of citrus canker disease on five varieties during 2017–18 and 2018–19

Five citrus varieties, i.e., Jaffa, Kagzi lime, Mayer lemon, Succari and Grapefruit were used for the determination of environmental factors conducive for the development of citrus canker. All environmental variables had positive significant correlation with citrus canker on all varieties during both years. The highest disease incidence (up to 55%) was recorded for Grapefruit under 37.2°C maximum temperature, while low disease incidence (7%) was observed on Jaffa under 37°C (Fig 4). Minimum disease incidence of 7% and less than 8% was noticed on Jaffa under 27.9°C minimum temperature (Fig 5). Jaffa showed 6.5% disease incidence during both years under 79.8% relative humidity as compared to disease incidence on Kagzi lime (18.9%), Mayer lemon (25.8%), Succari (40.5%) and Grapefruit (55.7%) (Fig 6). The similar variety Grapefruit showed 55.7% disease incidence 7.3 mm and 4.9 mm rainfall during 1^st^ and 2^nd^ year, respectively. Jaffa expressed relatively low disease incidence (<7%) (Fig 7). Disease incidence of less than 10% was recorded on Jaffa under 8 km/h wind speed during 2017 and 2018 (Fig 8). It was noticed that disease incidence increased from 8.5 to 55.7 and 8 to 55.4% on Grapefruit with rain splashes increasing, during both 2017–18 and 2018–19, respectively and same pattern was observed on all other varieties.

**Fig 4:** Relationship of maximum temperature with the development of citrus canker disease with during 2017–18 (A) and 2018–19 (B).

**Fig 5:** Relationship of minimum temperature with the development of citrus canker disease during 2017–18 (A) and 2018–19 (B).

**Fig 6:** Relationship of relative humidity with the development of citrus canker disease during 2017–18 (A) and 2018–19 (B).

**Fig 7:** Relationship of rainfall with the development of citrus canker disease during 2017–18 (A) and 2018–19 (B).

**Fig 8:** Relationship of wind speed with the development of citrus canker disease during 2017–18 (A) and 2018–19 (B).

## Discussion

Host susceptibility, pathogen virulence and favorable environmental conditions are necessary for disease development. Environmental factors like temperature, rainfall, wind speed, and relative humidity are crucial elements for different diseases [48, 49]. Sudden fluctuations in these environmental conditions can favor the development of diseases [50–52]. These climatic conditions play a significant role in resistance/susceptibility of plants against pathogens. They can also change the growth pattern, production, dissemination, infection, survival of pathogen and the interaction between the host and causal agent [53–55].

All environmental factors expressed significant positive correlation with all tested varieties/cultivars in the present study. The highest disease incidence was observed under 20–28°C and 30–38°C minimum and maximum temperature, 47–74% relative humidity, 8 km/h wind speed and 4 mm rainfall during both years. Predictive model based upon two years data was developed, Y = +24.02 + 0.5585 X_1_ + 0.2997 X_2_ + 0.3534 X_3_ + 3.590 X_4_ + 1.639 X_5_ (Y = disease incidence X_1_ = maximum temperature, X_2_ = minimum temperature, X_3_ = relative humidity, X_4_ = rainfall and X_5_ = wind speed). The R^2^ value of 97.5% expressed that that model is statistically appropriate and revealed that all these prescribed factors contributed positively towards the development of citrus canker. Results of present study are supported by several earlier studies [17, 20, 56, 57] reporting that temperature, high relative humidity and strong wind with rain splash play a crucial role in the development of citrus canker diseases. Numerous studies concluded that mild temperature, humidity and wind driven rain exhibited major effect on disease development [32, 33, 58].

Environmental conditions prevailing after the contact of pathogen with the plants can help greatly in the development of disease. Temperature greatly influenced the initiation and development of plant diseases. Various pathogens complete their life cycle and multiplied much rapidly during the favorable temperature [59, 60]. Different plant diseases and pathogens prefer different lower and higher temperatures. Some bacterial pathogens like *Pseudomonas* grow faster in the presence of low temperature, while others like *Xanthomonas* and *Ralstonia* grow much faster under high temperature. Temperature is also responsible in favoring and inhibiting the expression of certain genes, rapid production of pathogenesis related proteins involved in disease resistance and susceptibility by affecting the genetic machinery of host cells [61, 62].

In contemporary studies, temperature (maximum and minimum) relative humidity, strong wind with heavy rainfall gave significant correlation with citrus canker disease on maximum varieties. A strong interaction between disease development and increase in relative humidity was seen, which has been witnessed in earlier studies [63, 64]. Pathogen can spread up-to 50 km/h in the high wind speed and by reducing wind speed in orchards can reduced the dispersal of *Xcc* [65, 66]. Rainfall also expressed highly positive correlation with the development of disease. Incidence of canker disease was significantly increased with increasing in rainfall [35]. These results were supported by some recent studies [21, 67] reporting that temperature with other environmental factors had a major role in disease development. Disease index of citrus canker was highest under increased temperature and relative humidity during the month of July followed by month of August and September [68, 69]. High precipitation with sharp wind also contributed in the multiplication of bacteria. The incidence of citrus canker was greater when the rainy season started in the month of September [70, 71].

The winds also take part in the prevalence of diseases by spreading the pathogens, increasing the number of lesions and somehow by accelerating the drying of wet surfaces of the plants. It also facilitates bacteria in releasing spores and transferred form diseased portions to healthy ones. Results of the present study are also supported by an early study [72] indicating that wind becomes more drastic and lethal when it is accompanied by heavy rain, especially for citrus canker. These wind-blown rain splashes caused injuries on the surface of plants which help a number of bacteria and other pathogens to get entry into the plants [42]. Rainstorm during monsoon also increases the epidemics of various bacterial diseases in the presence of active source of inoculum and spread through strong winds [73].

## Conclusion

All the environmental variables, i.e., maximum, and minimum temperature, relative humidity, rainfall, and wind speed had significant positive correlation with citrus canker development on all varieties. Due to sudden fluctuations in the weather conditions, continuous monitoring of environmental variables is necessary for accurate prediction of citrus canker and its management. Installation of weather stations in major citrus growing areas would be helpful in risk assessment and forecasting systems in a specific area. Based on data collected from different areas, a Decian Support System can be developed for precise management of disease.

## Supporting information

S1 Dataset (XLSX)

## References

[1] LahlaliR, JaouadM, MoininaA, MokriniF, BelabessZ (2021) Farmers’ knowledge, perceptions, and farm-level management practices of citrus pests and diseases in Morocco. Journal of Plant Diseases and Protection: 1–14.

[2] PovedaJ, RoeschlinRA, MaranoMR, FavaroMA (2021) Microorganisms as biocontrol agents against bacterial citrus diseases. Biological Control 158: 104602.

[3] CuiX, LiuK, AttaS, ZengC, ZhouC, et al. (2021) Two Unique Prophages of ‘Candidatus Liberibacter asiaticus’ Strains from Pakistan. Phytopathology®: PHYTO-10-20-0454-SC. doi: 10.1094/PHYTO-10-20-0454-SC 33356428

[4] ArifM, Siddique AasiM, FarooqM, AliH, Ul IslamS, et al. (2017) Spatio-temporal distribution of the peach fruit fly, Bactrocera zonata (Diptera: Tephritidae) infesting citrus orchards at Sargodha, Pakistan. Acta Entomologica Sinica 60: 1457–1466.

[5] NoorizadehS, GolmohammadiM, BagheriA, BertacciniA (2021) Citrus industry: Phytoplasma-associated diseases and related challenges for Asia, America and Africa. Crop Protection: 105822.

[6] SamwelJ, MsogoyaT, TryphoneG, MtuiHD, BaltazariA, et al. (2021) Effects pre-harvest hexanal application on fruit market attributes of orange varieties grown in Eastern zone of Tanzania. The Journal of Horticultural Science and Biotechnology 96: 364–371.

[7] KumarKK, ArthursS (2021) Recent advances in the biological control of citrus nematodes: a review. Biological Control: 104593.

[8] DawoodMA, El BasuiniMF, ZaineldinAI, YilmazS, HasanM, et al. (2021) Antiparasitic and antibacterial functionality of essential oils: an alternative approach for sustainable aquaculture. Pathogens 10: 185. doi: 10.3390/pathogens10020185 33572193PMC7914417

[9] TangX, WangX, HuangY, MaL, JiangX, et al. (2021) Natural variations of TFIIAγ gene and LOB1 promoter contribute to citrus canker disease resistance in Atalantia buxifolia. PLoS genetics 17: e1009316. doi: 10.1371/journal.pgen.1009316 33493197PMC7861543

[10] LiuB, LaiJ, WuS, JiangJ, KuangW (2021) Endophytic bacterial community diversity in two citrus cultivars with different citrus canker disease resistance. Archives of Microbiology: 1–10. doi: 10.1007/s00203-021-02530-0 34406444

[11] IslamMN, AliMS, ChoiS-J, HyunJ-W, BaekK-H (2019) Biocontrol of citrus canker disease caused by Xanthomonas citri subsp. citri using an endophytic Bacillus thuringiensis. The plant pathology journal 35: 486. doi: 10.5423/PPJ.OA.03.2019.0060 31632223PMC6788417

[12] PengA, ChenS, LeiT, XuL, HeY, et al. (2017) Engineering canker‐resistant plants through CRISPR/Cas9‐targeted editing of the susceptibility gene Cs LOB 1 promoter in citrus. Plant biotechnology journal 15: 1509–1519. doi: 10.1111/pbi.12733 28371200PMC5698050

[13] MartinsPM, WoodTK, de SouzaAA (2021) Persister Cells Form in the Plant Pathogen Xanthomonas citri subsp. citri under Different Stress Conditions. Microorganisms 9: 384. doi: 10.3390/microorganisms9020384 33672822PMC7918609

[14] Klein-GordonJM, XingY, GarrettKA, AbrahamianP, ParetML, et al. (2021) Assessing Changes and Associations in the Xanthomonas perforans Population Across Florida Commercial Tomato Fields Via a Statewide Survey. Phytopathology®: PHYTO-09-20-0402-R.10.1094/PHYTO-09-20-0402-R33048630

[15] KhalidMS, KhalidS, FarooqA, ShafiqueM, AmjadA, et al. (2021) Characterization of Kinnow Mandarin fruit blemishes and tree-fruit-environment (TFE) profile in relation to various blemishes causal agents. Pure and Applied Biology. Vol. 10, Issue 4, pp1206–1216.

[16] DewdneyM, GrahamJ, RogersM (2016) Citrus canker. Florida Citrus Pest Management Guide, SP-43: 93–96.

[17] HallDG, GottwaldTR, BockCH (2010) Exacerbation of citrus canker by citrus leafminer Phyllocnistis citrella in Florida. Florida Entomologist 93: 558–566.

[18] BockC, CookA, ParkerP, GottwaldT, GrahamJ (2012) Short‐distance dispersal of splashed bacteria of Xanthomonas citri subsp. citri from canker‐infected grapefruit tree canopies in turbulent wind. Plant pathology 61: 829–836.

[19] DewdneyM, GrahamJ (2014) Florida Citrus Pest Management Guide: Citrus Canker (EDIS). The Institute of Food and Agricultural Sciences (IFAS) University of Florida 182.

[20] BockC, GrahamJH, GottwaldTR, CookAZ, ParkerPE (2010) Wind speed and wind-associated leaf injury affect severity of citrus canker on Swingle citrumelo. European journal of plant pathology 128: 21–38.

[21] GottwaldTR, GrahamJH (2021) Symptoms and Signs. Phytopathology News.

[22] ArifM, AttaS, BashirMA, KhanMI, HussainA, et al. (2021) The impact of Fosetyl-Aluminium application timing on Karnal bunt suppression and economic returns of bread wheat (Triticum aestivum L.). Plos one 16: e0244931. doi: 10.1371/journal.pone.0244931 33428646PMC7799839

[23] AbbasMF, RafiqM, Al-SadiAM, AlfarrajS, AlharbiSA, et al. (2021) Molecular characterization of leaf spot caused by Alternaria alternata on buttonwood (Conocarpus erectus L.) and determination of pathogenicity by a novel disease rating scale. Plos one 16: e0251471. doi: 10.1371/journal.pone.0251471 33984023PMC8118258

[24] ChakrabortyS, NewtonAC (2011) Climate change, plant diseases and food security: an overview. Plant pathology 60: 2–14.

[25] JuroszekP, Von TiedemannA (2011) Potential strategies and future requirements for plant disease management under a changing climate. Plant Pathology 60: 100–112.

[26] GillD (2013) Citrus canker: A serious bacterial disease. Louisiana Department of Agriculture and Forestry State of Louisiana USA.

[27] KhanMA, AbidM (2007) Effect of environmental conditions on citrus canker disease development. Pak J Phytopathol 19: 139–144.

[28] YanQ, WangN (2012) High-throughput screening and analysis of genes of Xanthomonas citri subsp. citri involved in citrus canker symptom development. Molecular plant-microbe interactions 25: 69–84. doi: 10.1094/MPMI-05-11-0121 21899385

[29] RybakM, MinsavageGV, StallRE, JonesJB (2009) Identification of Xanthomonas citri ssp. citri host specificity genes in a heterologous expression host. Molecular Plant Pathology 10: 249–262. doi: 10.1111/j.1364-3703.2008.00528.x 19236573PMC6640320

[30] ZhouX, HuX, LiJ, WangN (2015) A novel periplasmic protein, VrpA, contributes to efficient protein secretion by the type III secretion system in Xanthomonas spp. Molecular Plant-Microbe Interactions 28: 143–153. doi: 10.1094/MPMI-10-14-0309-R 25338144

[31] SecretariatI, GullinoM, AlbajesR, Al-JbooryI, AngelottiF, et al. (2021) Scientific review of the impact of climate change on plant pests. Scientific review of the impact of climate change on plant pests-A global challenge to prevent and mitigate plant pest risks in agriculture, forestry and ecosystems.

[32] RazaMM, KhanMA, AtiqM, BinyaminR, JavaidM (2014) Prediction of citrus canker epidemics generated through different inoculation methods. Archives of Phytopathology and Plant Protection 47: 1335–1348.

[33] Ting-shanY, YanZ, Chang-yongZ (2015) Research development of the differentiation and control of citrus bacterial canker disease. Acta Horticulturae Sinica 42: 1699.

[34] KumarP, DashyalMS, DoddarajuP, MetiBS, GirigowdaM (2021) Differential gene responses in different varieties of pomegranate during the pathogenesis of Xanthomonas axonopodis pv. punicae. 3 Biotech 11: 1–17. doi: 10.1007/s13205-020-02554-1 33927971PMC7981347

[35] AroraA, KaurS, RattanpalH, SinghJ (2013) Development of citrus canker in relation to environmental conditions. Plant Disease Research 28: 100–101.

[36] ChatterjeeS, HadiAS (2006) Regression analysis by example: John Wiley & Sons.

[37] GunstRF, MasonRL (2018) Regression analysis and its application: a data-oriented approach: CRC Press.

[38] HosmerDWJr, LemeshowS, SturdivantRX (2013) Applied logistic regression: John Wiley & Sons.

[39] KostS, RheinbachO, SchaebenH (2021) Using logistic regression model selection towards interpretable machine learning in mineral prospectivity modeling. Geochemistry: 125826.

[40] WilliamsLJ, AbdiH (2010) Fisher’s least significant difference (LSD) test. Encyclopedia of research design 218: 840–853.

[41] GottwaldTR, IreyM (2007) Post-hurricane analysis of citrus canker II: predictive model estimation of disease spread and area potentially impacted by various eradication protocols following catastrophic weather events. Plant Health Progress 8: 22.

[42] BockC, GrahamJ, GottwaldT, CookA, ParkerP (2010) Wind speed effects on the quantity of Xanthomonas citri subsp. citri dispersed downwind from canopies of grapefruit trees infected with citrus canker. Plant Disease 94: 725–736. doi: 10.1094/PDIS-94-6-0725 30754309

[43] SteelR (1997) Analysis of variance II: multiway classifications. Principles and procedures of statistics: A biometrical approach: 204–252.

[44] FerreiraDF (2019) SISVAR: A computer analysis system to fixed effects split plot type designs. Revista brasileira de biometria 37: 529–535.

[45] BockC, ParkerP, CookA, GottwaldT (2008) Visual rating and the use of image analysis for assessing different symptoms of citrus canker on grapefruit leaves. Plant Disease 92: 530–541. doi: 10.1094/PDIS-92-4-0530 30769647

[46] BockC, CookA, ParkerP, GottwaldT (2009) Automated image analysis of the severity of foliar citrus canker symptoms. Plant disease 93: 660–665. doi: 10.1094/PDIS-93-6-0660 30764402

[47] ElliottAC, HynanLS (2011) A SAS® macro implementation of a multiple comparison post hoc test for a Kruskal–Wallis analysis. Computer methods and programs in biomedicine 102: 75–80. doi: 10.1016/j.cmpb.2010.11.002 21146248

[48] NegiA (2015) Studies on characterization and management of Xanthomonas axonopodis pv. citri, the cause of citrus canker: GB Pant University of Agriculture and Technology, Pantnagar-263145 (Uttarakhand).

[49] KatkarM, RaghuwanshiK, ChimoteV, BorkarS (2016) Pathological, bio-chemical and molecular diversity amongst the isolates of Xanthomonas axonopodis pv. citri causing citrus canker in acid lime from different agro-climatic region of India. International Journal of Environment, Agriculture and Biotechnology 1: 238532.

[50] FerrareziRS, RodriguezK, SharpD (2020) How historical trends in Florida all‐citrus production correlate with devastating hurricane and freeze events. Weather 75: 77–83.

[51] FerrareziRS, QureshiJA, WrightAL, RitenourMA, MacanNP (2019) Citrus production under screen as a strategy to protect grapefruit trees from Huanglongbing disease. Frontiers in plant science 10: 1598. doi: 10.3389/fpls.2019.01598 31921247PMC6930270

[52] KadyampakeniDM (2020) Interaction of soil boron application with leaf B concentration, root length density, and canopy size of citrus affected by Huanglongbing. Journal of Plant Nutrition 43: 186–193.

[53] GhiniR, HamadaE, BettiolW (2008) Climate change and plant diseases. Scientia Agricola 65: 98–107.

[54] GraceMA, AchickT-FE, BonghanBE, BihME, NgoNV, et al. (2019) An overview of the impact of climate change on pathogens, pest of crops on sustainable food biosecurity. Int J Ecotoxicol Ecobiol 4: 114–119.

[55] SkendžićS, ZovkoM, ŽivkovićIP, LešićV, LemićD (2021) The Impact of Climate Change on Agricultural Insect Pests. Insects 12: 440. doi: 10.3390/insects12050440 34066138PMC8150874

[56] Jesus JuniorWC, Belasque JúniorJ, AmorimL, ChristianoRSC, ParraJRP, et al. (2006) Injuries caused by citrus leafminer (Phyllocnistis citrella) exacerbate citrus canker (Xanthomonas axonopodis pv. citri) infection. Fitopatologia Brasileira 31: 277–283.

[57] BockCH, GrahamJH, GottwaldTR, CookAZ, ParkerPE (2014) Effect of the duration of inoculum exposure on development of citrus canker symptoms on seedlings of Swingle citrumelo. European journal of plant pathology 138: 237–245.

[58] NeriFM, CookAR, GibsonGJ, GottwaldTR, GilliganCA (2014) Bayesian analysis for inference of an emerging epidemic: citrus canker in urban landscapes. PLoS Computational Biology 10: e1003587. doi: 10.1371/journal.pcbi.1003587 24762851PMC3998883

[59] Gómez ExpósitoR, De BruijnI, PostmaJ, RaaijmakersJM (2017) Current insights into the role of rhizosphere bacteria in disease suppressive soils. Frontiers in Microbiology 8: 2529. doi: 10.3389/fmicb.2017.02529 29326674PMC5741648

[60] RaaijmakersJM, PaulitzTC, SteinbergC, AlabouvetteC, Moënne-LoccozY (2009) The rhizosphere: a playground and battlefield for soilborne pathogens and beneficial microorganisms. Plant and soil 321: 341–361.

[61] ZandalinasSI, RiveroRM, MartínezV, Gómez-CadenasA, ArbonaV (2016) Tolerance of citrus plants to the combination of high temperatures and drought is associated to the increase in transpiration modulated by a reduction in abscisic acid levels. BMC plant biology 16: 1–16. doi: 10.1186/s12870-015-0700-5 27121193PMC4848825

[62] ZandalinasSI, BalfagónD, ArbonaV, Gómez‐CadenasA (2018) Regulation of citrus responses to the combined action of drought and high temperatures depends on the severity of water deprivation. Physiologia plantarum 162: 427–438. doi: 10.1111/ppl.12643 28902955

[63] ZandalinasSI, SalesC, BeltránJ, Gómez-CadenasA, ArbonaV (2017) Activation of secondary metabolism in citrus plants is associated to sensitivity to combined drought and high temperatures. Frontiers in plant science 7: 1954. doi: 10.3389/fpls.2016.01954 28119698PMC5220112

[64] Vives-PerisV, Gómez-CadenasA, Pérez-ClementeRM (2017) Citrus plants exude proline and phytohormones under abiotic stress conditions. Plant cell reports 36: 1971–1984. doi: 10.1007/s00299-017-2214-0 29038909

[65] IreyM, GottwaldTR, GrahamJH, RileyTD, CarltonG (2006) Post-hurricane analysis of citrus canker spread and progress towards the development of a predictive model to estimate disease spread due to catastrophic weather events. Plant Health Progress 7: 16.

[66] GottwaldT, GrahamJ, BockC, BonnG, CiveroloE, et al. (2009) The epidemiological significance of post-packinghouse survival of Xanthomonas citri subsp. citri for dissemination of Asiatic citrus canker via infected fruit. Crop Protection 28: 508–524.

[67] BehlauF, BelasqueJJr, Bergamin FilhoA, GrahamJ, LeiteRJr, et al. (2008) Copper sprays and windbreaks for control of citrus canker on young orange trees in southern Brazil. Crop Protection 27: 807–813.

[68] GrahamJ, JohnsonE, MyersM, YoungM, RajasekaranP, et al. (2016) Potential of nano-formulated zinc oxide for control of citrus canker on grapefruit trees. Plant disease 100: 2442–2447. doi: 10.1094/PDIS-05-16-0598-RE 30686171

[69] MichavilaG, AdlerC, De GregorioPR, LamiMJ, Caram Di SantoMC, et al. (2017) Pseudomonas protegens CS 1 from the lemon phyllosphere as a candidate for citrus canker biocontrol agent. Plant Biology 19: 608–617. doi: 10.1111/plb.12556 28194866

[70] ChristianoR, Dalla PriaM, JuniorWJ, ParraJ, AmorimL, et al. (2007) Effect of citrus leaf-miner damage, mechanical damage and inoculum concentration on severity of symptoms of Asiatic citrus canker in Tahiti lime. Crop Protection 26: 59–65.

[71] CanterosBI, GochezAM, MoschiniRC (2017) Management of citrus canker in Argentina, a success story. The plant pathology journal 33: 441. doi: 10.5423/PPJ.RW.03.2017.0071 29018307PMC5624486

[72] PkaniaKC, KrisA, GeertH, VennemanJ, KiplagatO, et al. (2014) Diversity Studies of Xanthomonas citri pv. malvacearum Strains Isolated from Cotton in Western Kenya Based on Rep PCR Analysis. African Journal of Education, Science and Technology 1: 142–149.

[73] Nawfal DagherT, Al-BayssariC, DieneSM, AzarE, RolainJ-M (2020) Bacterial infection during wars, conflicts and post-natural disasters in Asia and the Middle East: a narrative review. Expert review of anti-infective therapy 18: 511–529. doi: 10.1080/14787210.2020.1750952 32267179

